# Different Designs of Proximal Femoral Stems for Total Hip Arthroplasty: Mid-Term Clinical and Patient-Reported Functional Outcomes

**DOI:** 10.7759/cureus.19745

**Published:** 2021-11-19

**Authors:** Akhil Katakam, Shayan Hosseinzadeh, Tyler J Humphrey, Austin Collins, David Shin, Christopher M Melnic, Charles Bragdon, Hany S Bedair

**Affiliations:** 1 Orthopaedics, Massachusetts General Hospital, Harvard Medical School, Boston, USA

**Keywords:** promis, hoos, femoral stem design, total hip arthroplasty (tha), patient reported outcome measures

## Abstract

Introduction: A comprehensive comparison of the performance of different femoral stem geometries in total hip arthroplasty (THA) is yet to be described. The primary aim of this study was to evaluate objective and subjective outcome measures in primary THA with different femoral implant styles.

Methods: Stems were classified into the following five classes: cemented, conical, fit and fill, modular, and wedge. The objective outcomes of interest were the length of inpatient hospital stay (LOS), 90-day readmission rate, one-year revision rate, and two-year mortality rate. Preoperative and postoperative patient-reported outcome measures (PROMs), including hip disability and osteoarthritis outcome score (HOOS) - physical function shortform (HOOS-PS), patient-reported outcomes measurement information system physical function short form 10a (PROMIS PF-10a), and patient-reported outcomes measurement information system - short form - mental 10a (PROMIS M-10a) were recorded and compared between different classes.

Results: Patients with a wedge stem had a significantly lower LOS versus every other stem group, while patients with a cemented stem had the highest LOS, approximately twofold that of the wedge stem group. Accounting for potential confounders, the conical and fit and fill groups had a significantly higher two-year mortality rate than the wedge stem group. Fit and fill stems conferred a slight risk of revision THA at one-year compared to wedge stems. There was no significant difference in the rates of failure to achieve the minimal clinically important difference (MCID) for the PROMs.

Conclusion: Placement of wedge stems resulted in a significantly lower LOS compared to every other stem class and a lower mortality rate than the conical, fit and fill, and modular stems. As for the 90-day readmission, one-year revision, and the rates of failure to achieve the MCID for general or hip-specific PROMs, stem design had no meaningful effect.

## Introduction

Total hip arthroplasty (THA) is among the most commonly performed orthopaedic procedures, indicated in the management of hip arthritis for patients who have failed conservative management [1]. The surgery involves the removal of arthritic articular surfaces of the hip joint, which are then replaced by prosthetic hip components made of metal and polyethylene [2]. Assessment of THA outcomes may include objective outcomes such as length of stay (LOS), readmission rate, revision rate, and mortality [2-5]. In addition, patient-reported outcome measures, or PROMs, may be used to incorporate subjective patient assessments of their symptom state in the analysis of THA outcomes [6]. PROMs may vary in the domains that are assessed, for example, the PROMIS-10 physical (PROMIS PF-10a) and mental (PROMIS M-10a) global health scores aim to measure the overall physical and mental health of the patient, while a PROM such as the hip disability and osteoarthritis outcome score (HOOS) focuses on pain and function of the hip joint [7,8]. All of these aforementioned PROMs have been validated for responsiveness in measuring THA outcomes, and are used extensively in THA research [6,7]. One approach to interpreting PROM scores in the context of surgical intervention is to use the minimal clinically important difference (MCID) as a threshold for changes in PROM scores reflecting meaningful changes from preoperative to the postoperative symptom states for patients [9].

Many variations of prosthetic hip implants are currently in use with differences in materials, design rationales, and methods of fixation. Different implant types have been assessed with respect to performance and complication rates, such as the comparison of cemented and uncemented femoral stems and short-length femoral stems versus conventional-length femoral stems [10,11]. Although some arthroplasty registries and databases may report data on individual implant models, a comprehensive comparison of the performance of different femoral stem geometries has not yet been published in the literature. Moreover, it is unclear if a particular implant style may lead to higher rates of patients achieving MCID after THA.

The primary aim of this study is to evaluate objective and subjective outcome measures in primary THA with different femoral implant styles. Our first question was: are the objective measures of length of stay (LOS), 90-day readmission rate, one-year revision rate, and two-year mortality associated with different femoral implant styles in primary THA? Our second question was: are the subjective measures of achieving MCID on three different PROMs (HOOS, PROMIS PF-10a, PROMIS M-10a) affected by different femoral implant styles in primary THA?

## Materials and methods

This retrospective study was performed with Institutional Review Board approval using data from an arthroplasty registry within a regional network of hospitals supplemented with implant model data from the International Prostheses Library (IPL), a database of medical device information developed and maintained by the American Joint Replacement Registry (AJRR). The registry was queried for patients who had undergone primary total hip arthroplasty from June 2016 with at least two years of clinical follow-up.

Using these criteria, 7,732 THA patients were selected for analysis. The following demographic variables were obtained from the registry and through a chart review: age, body mass index (BMI), Charlson comorbidity index (CCI), discharge disposition, hospital, sex, readmission within 90 days, revision within one year, mortality within two years, and diagnoses of major depressive disorder, type II diabetes, chronic obstructive pulmonary disorder (COPD), arrhythmia, or hypertension. Stem manufacturer and stem model names were also obtained from the registry. Stems were classified into the following five classes: cemented, conical, fit and fill, modular, and wedge. A full list of stem manufacturers, models, and classifications can be found in Table 1.

**Table 1:** Summary of Stem Manufacturers, Model Names, and Classifications

Manufacturer	Model Name	Class	Frequency (n=7,732)
Corin	Metafix	Wedge	20 (0.26%)
Corin	Mini Hip System	Wedge	53 (0.69%)
Corin	TriFit	Wedge	17 (0.22%)
DePuy	Corail	Wedge	1337 (17.29%)
DePuy	Reclaim	Modular	2 (0.03%)
DePuy	S-Rom	Modular	162 (2.10%)
DePuy	Summit	Fit and Fill	653 (8.45%)
DePuy	Tri-Lock	Wedge	155 (2.00%)
Osteonics	Omnifit	Cemented	1 (0.01%)
Smith & Nephew	Anthology	Wedge	190 (2.46%)
Smith & Nephew	Synergy	Fit and Fill	57 (0.74%)
Stryker	Accolade C	Wedge	1 (0.01%)
Stryker	Accolade II	Wedge	1552 (20.07%)
Stryker	Exeter V40	Cemented	38 (0.49%)
Stryker	Omnifit	Cemented	30 (0.39%)
Stryker	Restoration	Modular	6 (0.08%)
Stryker	Secur-Fit	Fit and Fill	344 (4.45%)
Zimmer Biomet	Arcos	Modular	4 (0.05%)
Zimmer Biomet	Avenir	Wedge	5 (0.06%)
Zimmer Biomet	Echo	Wedge	130 (1.68%)
Zimmer Biomet	Echo BiMetric Microplasty	Wedge	151 (1.95%)
Zimmer Biomet	Taperloc Microplasty	Wedge	701 (9.07%)
Zimmer Biomet	Taperloc	Wedge	985 (12.74%)
Zimmer Biomet	CPT	Cemented	3 (0.04%)
Zimmer Biomet	M/L Taper	Wedge	778 (10.06%)
Zimmer Biomet	VerSys	Fit and Fill	311 (4.02%)
Zimmer Biomet	Wagner	Conical	46 (0.59%)

The objective outcomes of interest were the length of inpatient hospital stay, 90-day readmission rate, one-year revision rate, and two-year mortality rate. Preoperative and postoperative PROMs, including HOOS-PS, PROMIS PF-10a, and PROMIS M-10a were recorded. Preoperative PROMs were included for analysis if they were completed within six months prior to THA. Postoperative PROMs were included if they were completed between six months and two years following THA, these intervals for both preoperative and postoperative PROMs have been justified in similar studies [12-15]. There were 1692 patients who completed both preoperative and postoperative PROMs who were included for MCID analysis. For this cohort of patients, the primary outcomes of interest were failure to achieve the MCID on the HOOS-PS, PROMIS PF-10a, and PROMIS M-10a. A change of PROM score from pre- to post-THA of 9.3 (HOOS-PS), 4.1 (PROMIS PF-10a), and 3.7 (PROMIS M-10a) were determined as the threshold for achieving MCID using the distribution-based method, a validated method that sets the MCID threshold as one-half of the standard deviation of PROM change from preoperative to postoperative states across all patients [16-18]. If the difference between the preoperative to postoperative PROM for a patient was higher than the MCID threshold, he or she was classified as having achieved the MCID.

Statistical analysis

Frequencies and proportions were used to describe categorical variables and means, and standard deviations (SD) were used to describe continuous variables. To assess the association between stem style and objective outcomes, univariate analysis was first performed with all collected variables and each outcome. The relationship between categorical variables and each objective outcome was analyzed with a chi-squared test of independence; continuous variables were evaluated with Student’s t-tests. Variables that were associated (defined by p<0.2) with an outcome were included in a multivariable logistic or linear regression model to assess for potential confounders. For all variables analyzed in multivariable logistic regression, odds ratios (OR), 95% confidence intervals (CI), and p-values were reported. For variables analyzed in multivariable linear regression, β coefficients, 95% CIs, and p-values were reported. For patients who completed both preoperative and postoperative PROMs, differences in the means were compared using analysis of variance (ANOVA) and Student’s t-tests. The Tukey post-hoc test was used to determine which stem styles were statistically different with respect to MCID achievement. Statistical significance was defined as p<0.05. Post-hoc power analyses were performed for comparisons failing to achieve significance to determine the likelihood of a type II error. All statistical analyses were performed using R (The R Foundation, Vienna, Austria) and RStudio (RStudio, Boston, MA).

## Results

Mean age, BMI, and CCI across the entire patient cohort were 64.9 years (SD 11.8), 29.0 kg/m2 (SD 5.7), and 0.8 (SD 1.4), respectively. Five patients were discharged to a custodial care facility, 412 patients were discharged home without services, 5882 patients were discharged to home health care, six patients were discharged to hospice care, 10 patients were discharged to a long-term care facility, 234 patients were discharged to a rehabilitation facility, three were discharged to a short-term hospital, and 1,180 were discharged to a skilled nursing facility. The entire study cohort was composed of 3,592 (46.5%) males.

There were 72 (0.9%), 46 (0.6%), 1365 (17.7%), 174 (2.3%), and 6075 (78.6%) cemented, conical, fit and fill, modular, and wedge stem styles used, respectively. Demographics stratified by stem style are shown in Table 2. Age (77.0 years vs. 64.8 years; p<0.001) and CCI (2.0 vs. 0.8; p<0.001) were significantly higher in the cemented stem group compared to all other groups. BMI was significantly lower in the cemented stem group compared to the fit and fill (26.8 kg/m2 vs. 29.4 kg/m2; p<0.001), modular (26.8 kg/m2 vs. 29.6 kg/m2; p<0.001), and wedge (26.8 kg/m2 vs. 28.9 kg/m2; p<0.001) groups. The cemented stem group had the longest mean LOS compared with all other groups (5.2 days vs. 2.6 days; p<0.001). The fit and fill group also had a significantly greater LOS than the modular (3.2 days vs. 2.7 days; p=0.006) and wedge (3.2 days vs. 2.4 days; p<0.001) groups. The cemented stem group had the highest 90-day readmission rate (20.8%), whereas the conical stem class had the lowest rate (4.3%; p=0.013). The conical stem class had the highest two-year mortality rate (4.3%) while the wedge stem class had the lowest two-year mortality rate (0.6%; p=0.001); however, this difference was based on two mortalities in the conical stem class. There was a trend towards increased one-year revisions in the wedge class compared with the other classes; however, this difference was not significant and only based on two events in the wedge class (4.3% versus 2.0%; p=0.031).

**Table 2:** Demographic Summary of Collected Variables Stratified by Stem Design BMI: body mass index, CCI: Charlson comorbidity index, COPD: chronic obstructive pulmonary disease *Male sex versus female sex

Demographics	Cemented (n=72)	Conical (n=46)	Fit and Fill (n=1365)	Modular (n=174)	Wedge (n=6075)	p-value
Age	77.0±11.3	46.6±19.1	67.5±11.7	59.5±14.3	64.5±11.4	<0.001
BMI	26.8±6.8	28.3±5.6	29.4±6.0	29.6±5.4	28.9±5.6	<0.001
CCI	2.0±2.0	0.6±1.1	1.0±1.5	0.5±1.1	0.8±1.3	<0.001
Discharge Disposition						
Custodial Care Facility	4 (5.55%)	0 (0%)	1 (0.07%)	0 (0%)	0 (0%)	<0.001
Home or Self-Care	1 (1.38%)	5 (10.86%)	53 (3.88%)	36 (20.68%)	317 (5.31%)	<0.001
Home-Health Care Svc	13 (18.05%)	33 (71.73%)	957 (70.10%)	109 (62.64%)	4770 (78.51%)	<0.001
Hospice	0 (0%)	0 (0%)	0 (0%)	0 (0%)	6 (0.09%)	0.802
Long-term Care	0 (0%)	0 (0%)	3 (0.21%)	0 (0%)	7 (0.11%)	0.855
Rehabilitation Facility	13 (18.05%)	0 (0%)	65 (4.76%)	10 (5.74%)	146 (2.40%)	<0.001
Short-term Hospital	0 (0%)	0 (0%)	1 (0.07%)	0 (0%)	2 (0.03%)	0.965
Skilled Nursing Facility	41 (56.94%)	8 (17.39%)	285 (20.87%)	19 (10.91%)	827 (13.61%)	<0.001
Hospital (deidentified)						
A	16 (22.22%)	14 (30.43%)	439 (32.16%)	116 (66.67%)	1407 (23.16%)	<0.001
B	12 (16.67%)	4 (8.69%)	185 (13.55%)	9 (5.17%)	761 (12.52%)	0.020
C	23 (31.94%)	15 (32.61%)	200 (14.65%)	8 (4.59%)	1770 (29.13%)	<0.001
D	0 (0%)	0 (0%)	83 (6.08%)	0 (0%)	0 (0%)	<0.001
E	2 (2.77%)	0 (0%)	343 (25.12%)	3 (1.72%)	251 (4.13%)	<0.001
F	19 (26.38%)	13 (28.26%)	115 (8.42%)	38 (21.83%)	1886 (31.04%)	<0.001
Male Sex*	12 (16.67%)	18 (39.13%)	554 (40.58%)	117 (67.24%)	2891 (47.58%)	<0.001
Diabetes	12 (16.67%)	2 (4.34%)	120 (8.79%)	2 (1.14%)	396 (6.51%)	<0.001
Depression	9 (12.50%)	7 (15.21%)	191 (13.99%)	20 (11.49%)	713 (11.73%)	0.215
COPD	9 (12.50%)	3 (6.52%)	49 (3.58%)	2 (1.14%)	141 (2.32%)	<0.001
Arrhythmia	21 (29.16%)	0 (0%)	135 (9.89%)	13 (7.47%)	488 (8.03%)	<0.001
Hypertension	53 (73.61%)	9 (19.56%)	690 (50.54%)	51 (29.31%)	2578 (42.43%)	<0.001
Length of Stay	5.2	3.1	3.2	2.7	2.4	<0.001
90-day Readmission	15 (20.8%)	2 (4.3%)	140 (10.3%)	18 (10.3%)	474 (7.8%)	<0.001
1-year Revision	1 (1.4%)	2 (4.3%)	41 (3.0%)	2 (1.1%)	108 (1.8%)	0.031
2-year Mortality	2 (2.8%)	2 (4.3%)	31 (2.3%)	3 (1.7%)	34 (0.6%)	<0.001

Table 3 shows the multivariable linear regression model of variables associated with LOS. The wedge stem group experienced a significantly lower LOS compared to every other stem class. Notably, the cemented stem class suffered 2.07 days of increased hospital stay compared to the wedge stem class. Table 4 demonstrates that the 90-day readmission rate was similar between stem classes when accounting for confounders. Based on current information on variables associated with 90-day readmission rate, 1 - beta = 0.89, indicating the sample size was adequately powered at 89% to detect differences between the groups.

**Table 3:** Multivariable Linear Regression of Candidate Variables to Predict Length of Stay BMI: body mass index, CCI: Charlson comorbidity index, COPD: chronic obstructive pulmonary disease *Male sex versus female sex

Variables	β Coefficient	95% Confidence Interval	P-value
Age	0.02	0.00-0.02	<0.001
BMI	0.01	0.00-0.02	0.001
CCI	0.20	0.18-0.21	<0.001
Male Sex*	-0.29	-0.33- -0.25	<0.001
Type II Diabetes	0.11	0.01-0.20	0.241
MDD	0.11	0.04-0.18	0.094
COPD	0.84	0.70-0.98	<0.001
Arrhythmia	0.39	0.31-0.47	<0.001
Hypertension	-0.05	-0.10-0.00	0.294
Stem Type			
Wedge	Reference	Reference	Reference
Cemented	2.07	1.85-2.29	<0.001
Conical	0.98	0.70-1.26	<0.001
Fit and Fill	0.63	0.57-0.69	<0.001
Modular	0.45	0.31-0.59	0.001

**Table 4:** Multivariable Logistic Regression of Candidate Variables to Predict 90-Day Readmission Rate BMI: body mass index, CCI: Charlson comorbidity index, COPD: chronic obstructive pulmonary disease, LOS: length of stay, MDD: major depressive disorder

Variables	Odds Ratio	95% Confidence Interval	P-value
Age	1.01	1.00-1.02	0.057
CCI	1.11	1.05-1.18	<0.001
LOS	1.15	1.11-1.20	<0.001
Type II Diabetes	0.93	0.67-1.25	0.625
MDD	1.55	1.24-1.92	<0.001
COPD	1.11	0.71-1.68	0.642
Arrhythmia	1.10	0.83-1.43	0.504
Hypertension	1.25	1.04-1.49	0.018
Stem Type			
Wedge	Reference	Reference	Reference
Cemented	1.48	0.76-2.69	0.224
Conical	0.49	0.08-1.76	0.360
Fit and Fill	1.10	0.89-1.35	0.370
Modular	1.45	0.85-2.34	0.148

Table 5 shows that the fit and fill stem group had a significantly higher rate of revision THA at one-year (OR 1.56; 95% CI 1.07-2.24) compared to the wedge stem group. Conical (OR 11.22; 95% CI 1.62-44.25) and fit and fill (OR 3.11; 95% CI 1.84-5.23) stem groups were found to have a two-year mortality rate significantly higher than the wedge stem group (Table 6).

**Table 5:** Multivariable Logistic Regression of Candidate Predictors to One-Year THA Revision Rate BMI: body mass index, CCI: Charlson comorbidity index, LOS: length of stay, MDD: major depressive disorder

Variables	Odds Ratio	95% Confidence Interval	P-value
BMI	1.03	1.00-1.05	0.035
CCI	1.07	0.96-1.18	0.212
LOS	1.06	1.02-1.11	0.004
MDD	1.68	1.10-2.48	0.013
Stem Type			
Wedge	Reference	Reference	Reference
Cemented	0.60	0.03-2.82	0.617
Conical	2.34	0.37-7.89	0.251
Fit and Fill	1.56	1.07-2.24	0.018
Modular	0.63	0.10-2.01	0.519

**Table 6:** Multivariable Logistic Regression of Candidate Predictors to One-Year Mortality Rate BMI: Body mass index, CCI: Charlson comorbidity index, COPD: chronic obstructive pulmonary disease, LOS: length of stay, MDD: major depressive disorder

Variables	Odds Ratio	95% Confidence Interval	P-value
Age	1.04	1.01-1.06	0.003
BMI	0.95	0.90-0.99	0.031
CCI	1.18	1.02-1.34	0.021
LOS	1.15	1.09-1.22	<0.001
MDD	1.78	0.94-3.18	0.061
COPD	1.53	0.56-3.59	0.366
Arrhythmia	0.89	0.39-1.82	0.761
Hypertension	1.00	0.58-1.73	0.996
Stem Type			
Wedge	Reference	Reference	Reference
Cemented	1.23	0.18-4.79	0.798
Conical	11.22	1.62-44.25	0.003
Fit and Fill	3.11	1.84-5.23	<0.001
Modular	4.08	0.96-11.76	0.023

The rates of MCID achievement across the three PROMs collected are reported in Table 7, stratified by stem style. From the original cohort, seven (9.7%) cemented stem, seven (15.2%) conical stem, 230 (16.8%) fit and fill stem, 50 (28.7%) modular stem, and 1398 (23.0%) wedge stem patients completed preoperative and postoperative PROMs. The rates of failure to achieve the MCID for the HOOS-PS (p=0.187), PROMIS 10-Physical (p=0.593), and PROMIS 10-Mental (p=0.569) were similar between groups. Based on the current numbers of completed PROMs, this sample size may not be adequately powered to detect differences across all the groups (1 - beta = 0.63). This was mainly due to the number of reported PROMs in the cemented and conical groups. If the two groups with the smallest sample size (cemented and conical) are excluded from the MCID analysis, the power of the comparison between the three remaining groups is 83%. Based on this, it appears that a difference did not exist in the rates of achieving MCID between the wedge, fit, and fill or modular stems groups.

**Table 7:** Failure of MCID Achievement Across HOOS-PS, PROMIS PF-10a, and PROMIS M-10a Stratified by Stem Design HOOS-PS: Hip disability and osteoarthritis outcome score (HOOS) – physical function shortform, PROMIS PF-10a: The patient-reported outcome measurement information system physical function short form 10a, PROMIS M-10a: patient reported outcomes measurement information system - short form - mental 10a

Failure of MCID Achievement	Cemented (n=7)	Conical (n=7)	Fit and Fill (n=230)	Modular (n=50)	Wedge (n=1398)	p-value
HOOS-PS	3 (42.9)	3 (42.9)	40 (17.4)	8 (16.0)	247 (17.7)	0.187
PROMIS PF-10a	2 (28.6)	2 (28.6)	76 (33.0)	14 (28.0)	387 (27.7)	0.593
PROMIS M-10a	2 (28.6)	5 (71.4)	132 (57.4)	28 (56.0)	790 (56.5)	0.569

## Discussion

In summary, these findings show a few differences in clinical outcomes of different stem designs. Notably, those patients who had a wedge stem had a significantly lower LOS compared to every other stem group, while those with a cemented stem had the highest LOS, approximately twofold that of the wedge stem group. Even when accounting for potential confounders such as CCI and age, the conical and fit and fill groups were found to have a significantly higher two-year mortality rate than the wedge stem group. The conical stem group's increased odds for two-year mortality, as seen in the +11.22 odds ratio, may be exaggerated due to the relatively low sample size of 46 patients in the group with two mortalities reported. There were no significant differences between the 90-day readmission rate between stem groups when accounting for the confounders. Fit and fill stems conferred a slight risk of revision THA at one year compared to wedge stems. With the available numbers, we could not detect any significant difference in the rates of failure to achieve the MCID for the measured PROMs.

Over the past five decades, the femoral stem design of THA implants has changed in response to identified needs such as improved longevity, improved materials, and ease of use, and now there exist many viable options for an orthopaedic surgeon to choose [19]. The stem design and shape of the prosthesis is known to be an important factor for determining the stress distribution of the proximal femur, which could potentially have a role in better surgical outcomes [20]. While cemented stems can yield excellent outcomes and have the potential to establish an efficient metaphyseal-loading regimen, one of the main reasons for the introduction of the cementless stems was to improve outcomes in younger, more active patients [21,22]. Of note, the uncemented femoral stem has shown lower rates of aseptic loosening compared to the cemented stems [21]. Many different cementless stem designs have been developed, such as the fit and fill stems, which aim to fill the metaphysis in both sagittal and coronal planes by contacting most of the metaphysis, while the tapered wedge femoral stems are designed for a more congruent cortical fit in the coronal plane to achieve a better proximal mediolateral fixation [23,24]. Wedging a tapered design stem into the femur to achieve stability can efficiently decrease the prosthesis stiffness compared to a cylindrical stem with backbone rubbing fixation [25]. Conical stems, on the other hand, were designed to provide axial and diaphyseal rotational stability without version constraint, and modular components were designed to decouple the metaphyseal and diaphyseal geometries [26,27].

Previous studies often focus on the comparison of two different specific stem designs or the comparison of two different stems belonging to the same design class but produced by different manufacturers [18,28,29]. This study serves as the first retrospective multicenter study to investigate differences in clinical and patient-reported outcomes based on the femoral stem design family. A shorter LOS and an increased rate of discharge to home are cost-effective approaches [28]. While our findings of a higher LOS and similar two-year mortality, 90-day readmission, and one-year revision rates of cemented stems compared to wedge stems may appear to be in contrast to a previous study by Chammout et al., which was performed specifically on displaced femoral neck fractures in the elderly; the conclusions from our study show consistency with the body of literature using a broader patient population that helps to ensure generalizability by better representing the target population [29].

Patients across all stem designs were found to fail to achieve the MCID for the HOOS-PS, PROMIS 10 physical, and PROMIS 10 mental with similar frequency. This finding would indicate that stem design alone does not influence MCID achievement for general or hip-specific PROMs. Limited PROM completion rate among this cohort prohibited multivariable regression analysis, which may have revealed subtle yet pertinent differences between stem performance.

There are some limitations to our study. The main limitation is that even though we were adequately powered to compare different groups with regards to clinical outcomes, we had a relatively small sample size for the PROMs comparison; therefore, orthopaedic surgeons should be cautious when considering the results of the failure to achieve the MCID in the cemented and conical groups as this element on investigation may be lacking the power to detect meaningful differences. Future studies should attempt to conduct similar analyses on a larger patient population with available PROMs. However, based on current PROM results, at least it can be concluded that there is no difference in PROMs between the most popular stem designs. The retrospective and cross-sectional nature of this study are among other limitations that hinder our ability to assess the exposure and outcomes. For example, the choice of the stem was made by the operating surgeon, and the details of why a specific stem may have been chosen are not available.

## Conclusions

Reflecting the standard of care in the United States, the present analysis found that wedge stems result in a significantly lower LOS compared to every other stem class, and a lower mortality rate than the conical, fit and fill, and modular stem classes. As for the 90-day readmission, one-year revision, and the rates of failure to achieve the MCID for general or hip-specific PROMs, stem design had no meaningful effect. Future prospective studies should be conducted to validate these findings.
